The article "Mechanistic attributes of S100A7 (psoriasin) in resistance of anoikis resulting tumor progression in squamous cell carcinoma of the oral cavity" was retracted in 2021. Reason: concerns about the images.

# Mechanistic attributes of S100A7 (psoriasin) in resistance of anoikis resulting tumor progression in squamous cell carcinoma of the oral cavity

**DOI:** 10.1186/s12935-015-0226-9

**Published:** 2015-07-29

**Authors:** Kaushik Kumar Dey, Siddik Sarkar, Ipsita Pal, Subhasis Das, Goutam Dey, Rashmi Bharti, Payel Banik, Joygopal Roy, Sukumar Maity, Indranil kulavi, Mahitosh Mandal

**Affiliations:** School of Medical Science and Technology, Indian Institute of Technology, Kharagpur, 721302 West Bengal India; Dr Rafi Ahmed Dental College and Hospital, Kolkata, 700014 West Bengal India; Calcutta Medical College, Kolkata, 700073 West Bengal India; Bankura Sammilani Medical College, Bankura, 722101 West Bengal India

**Keywords:** Psoriasin, S100A7, Anoikis, Squamous cell carcinoma, Cell proliferation, Apoptosis

## Abstract

**Background:**

Squamous cell carcinoma of the oral cavity (SCCOC) is the dominant origin of cancer associated mortality. Previous findings by our study reported that acquisition of anoikis resistance has a significant role in tumor progression of oral cavity. Several genes were over-expressed in anoikis-resistant cells under detached conditions which we confirmed earlier by microarray. Normal oral squamous epithelia grow adherent to a basement membrane, and when detached from the extracellular matrix, undergoes programmed cell death. The acquisition of anoikis-resistance is crucial phenomena in oral tumor advancement. In the current study, we have identified S100A7 expression as contributing factor for anoikis resistance and tumorigenicity in human oral cancer cells. Further, we have explored that elevated S100A7 expression in anoikis-sensitive oral keratinocytes and cancer cells reshape them more resistant to anoikis and apoptosis inducers via activation of cellular intrinsic and extrinsic avenue.

**Methods:**

A subset of human cancer cell lines TU167, JMAR, JMARC39, JMARC42 and MDA-MB-468 were utilized for the generation of resistant stable cell lines. Further, immunohistochemistry, western blot and immunoprecipitation, assays of apoptosis, soft agar assay, orthotopic animal model and signaling elucidation were performed to establish our hypothesis.

**Results:**

S100A7 gene is found to be responsible for anoikis resistance and tumorigenicity in human oral cancer cells. We have observed up-regulation of S100A7 in anoikis resistant cell lines, orthotropic model and patients samples with head and neck cancer. It is also noticed that secretion of S100A7 protein in conditioned medium by anoikis resistant head & neck cancer cell and in saliva of head and neck cancer patients. Up-regulation of S100A7 expression has triggered enhanced tumorigenicity and anchorage-independent growth of cancer cells through Akt phosphorylation leading to development of aniokis resistance in head and neck cancer cells.

The article "Mechanistic attributes of S100A7 (psoriasin) in resistance of anoikis resulting tumor progression in squamous cell carcinoma of the oral cavity" was retracted in 2021. Reason: concerns about the images.

**Conclusions:**

These data have led us to conclude that S100A7 is the major contributing factor in mediating anoikis-resistance of oral cancer cells and local tumor progression, and S100A7 might be useful as diagnostic marker for early detection of primary and recurrent squamous cell cancer.

## Background

Cells undergo anchorage-independent cell death or an anoikis, as they separate and move towards the epithelial surface [1, 2]. Anoikis has a specific kind of physical characteristics similar to apoptosis, and it plays a crucial role in maintenance of normal tissue homeostasis and cell replacement [2]. Anoikis occurs due to the inappropriate or faulty cellular interaction between Cell and ECM that might lead to the prevention of detached cells to the improper location. The current knowledge suggested that keratinocytes underwent anoikis when these normal cells failed to attach to ECM [3]. Anoikis has a dominant involvement in the safeguard mechanisms of epithelial cells when they are in adherent culture, depending upon the interaction with ECM proteins. Due to anoikis resistance, some oral cavity cancer cell lines can grow in suspension due to the altered regulation of integrin and E-cadherin directed survival signaling [4, 5].

Anchorage-independent cell growth is an important physiological process for cancer development. To assess the tumorigenicity, the unique property of tumor cells to grow in soft agar was considered as an in vitro test in immunosuppressed animals [6]. During anoikis cells are detached from the ECM by mechanical forces or some other means to undergo apoptosis by extrinsic and intrinsic pathways. Failure to undergo anchorage-independent cell growth can be as an important hallmark of cancer owing to its property of invading through blood vessels and lymphatic stream. In order to support this fact, there are evidences that the passage of non-oncogenesis monkey kidney epithelial cells in suspension culture formed an anoikis-resistant line which leads to the generation of hypodermic tumors in nude mice [7]. Moreover, melanoma cell suspension culture exhibited anoikis resistance and metastasis, when administered through tail veins of mice [8]. While these earlier findings are supportive of our hypothesis, the correlation of in vitro anoikis resistance and metastasis potential has not been yet confirmed in an orthotropic in vivo tumor model. Literature suggested the involvement of TrkB protein in regulation of metastasis by screening of anoikis. In this current study, suitable experimental design and tumor model were developed to prove our hypothesis.

The article "Mechanistic attributes of S100A7 (psoriasin) in resistance of anoikis resulting tumor progression in squamous cell carcinoma of the oral cavity" was retracted in 2021. Reason: concerns about the images.

Psoriasin (S100A7), which belongs to S100 gene family [9], was first isolated from psoriasis affected skin [10]. It is an 11.4 kDa secretary protein, often responsible for inflammatory responses in the skin [11, 12]. Furthermore, altered keratinocyte differentiation in skin was observed [13, 14], and the differential expression of psoriasin was noted in squamous cell cancer (SCC) of bladder [15] and in breast carcinoma [16, 17]. Intensive studies revealed that increasing expression of psoriasin was well associated with early development of oncogenesis. Psoriasin was found to be up regulated in ductal carcinoma, but the expression of this protein was relatively low in adjacent invasive carcinoma [17]. The altered expression of psoriasin was associated with epithelial cell differentiation. S100A2 and S100A4, member of S100 gene family were found to be deregulated in breast cancer [18, 19]. Distinct changes in the expression profile of psoriasin were also noticed in benign tumors and high-grade DCIS [17, 20]. Altered expression of psoriasin also appeared to be associated with poor prognosis in several invasive tumor predominantly in ERα-ve and ERß-ve tumors [21]. Previous studies suggested that unlike the other category of S100 proteins counterpart, here psoriasin expression is generally controlled to the epithelial part of skin, breast, and bladder [11, 15, 21–23]. In hyperplasia and dysplasia mediated pathological conditions, the expression of psoriasin was relatively low in normal epithelial cells whereas it was mostly up-regulated in keratinocytes in the epidermis. Earlier report revealed that functional activity of psoriasin is regulated by a small cluster of gene. Serial analysis of gene expression (SAGE) profiling demonstrated that above gene population is significantly up-regulated in actinic keratosis compared to normal skin [13]. Only some of the genes, like psoriasin, were being expressed in the ‘epithelial differentiation complex’ region on chromosome 1q21 [24]. It was observed that the main cellular transformation behind invasive phenomena is dedifferentiation that is involved as an integral part of this process [25]. Several important factors were found to participate in controlling the regulation of psoriasin. Vitamin A derived metabolite retinoic acid included among these factors, which was found to be closely associated with the control of squamous cell differentiation [26]. Psoriasin regulating factors include irradiation by UV, calcium and altered cell attachment to the skin [26–30] and various physiological factors such as confluency, growth factor deprivation and loss of cellular attachment in breast epithelial cells [16, 20]. Further evidences confirmed that cell stress due to UV radiation promotes activation of AP-1 transcription factor complex mediated by c-Jun/JNK pathway [31]. It was noticed that skin tumorigenesis, progression, and invasion are caused due to the stimulation of the AP-1 pathway [32]. Our study is trying to establish the importance of psoriasin in anoikis resistance and head and neck cancer tumor progression.

The article "Mechanistic attributes of S100A7 (psoriasin) in resistance of anoikis resulting tumor progression in squamous cell carcinoma of the oral cavity" was retracted in 2021. Reason: concerns about the images.

## Results and discussion

### Identification of psoriasin (S100A7) as a regulatory gene

In an attempt to recognize genes whose appearance might be modulated in the human head and neck cancer cells, we have used microarray techniques. Initially, two cell lines: TU167 (less invasive) and JMAR (highly invasive) were cultured at both attach or detached condition for 24 and 48 h, total RNA was isolated, and cDNA probes were prepared using reverse transcription. Later, sequencing and comparison of the cDNA revealed that it was found to be 100% identical to human S100A7 [33]. To determine the expression of S100A7, cells were grown in suspension for 24 and 48 h, and the protein expressions were evaluated by western blot. As shown in Fig. 1a, S100A7 protein expression was up-regulated during detachment of JMAR C39 and JMAR C42 anoikis resistant cell line (soft agar clone derived from JMAR) and not in TU167, anoikis sensitive cell line indicating that S100A7 is one of the up-regulated genes responsible for anoikis resistance and tumor progression. S100A7 level was also observed to be up-regulated during anoikis in JMAR cells as shown by immunofluorescence microscopy (Fig. 1b). Further, TUNEL (Terminal deoxynucleotidyl transferase dUTP nick end labelling) assays were performed which shows increasing number of anoikis resistance cells (Fig. 1c). In the direction of confirmation of S100A7 gene was controlled by anoikis in HNSCC cells, regulation of the S100A7 gene expression was verified by experiments involving Northern blot analysis (Fig. 1d) showing the up-regulation of S100A7 mRNA in JMAR, JMARC39 (another soft agar clones derived from JMAR) and JMAR C42 during detached condition.

**Fig. 1:** Up-regulation of S100A7 protein and mRNA during detachment of anoikis resistant cell lines and in orthotopic mice model. **a** Both the attached and detached at different time points of cell lysates of TU167 and JMAR were analyzed by western blot for S100A7. β-actin was used as a loading control. **b** Detection of S100A7 in JMAR detached cells by immunofluorescence after staining with anti-S100A7. **c** TUNEL (Terminal deoxynucleotidyl transferase dUTP nick end labelling) assays were performed to study increasing anoikis resistance cells. **d** Northern blot showing expression of S100A7 mRNA in TU167 and various clones of JMAR in both attached and detached condition for indicated time intervals. **e** IHC of S100A7 expression for FFPE tumor sections of mice generated from orthotopic injection of TU167 and JMAR cell lines.

The article "Mechanistic attributes of S100A7 (psoriasin) in resistance of anoikis resulting tumor progression in squamous cell carcinoma of the oral cavity" was retracted in 2021. Reason: concerns about the images.

### Expression of the S100A7 in an orthotopic tumor model of squamous cell oral cancer

On the way to assess the property of tumor progression due to the selection for anoikis resistance, we have studied in vivo orthotopic tumor model with both the cells [26]. In the consequent experiment, TU167 or JMAR cells (5 × 10^5^) were injected in the tongues of the mutant (the nude) mice, which lead to tumor formation and weight loss in the animals. The development of tumors was also observed in both the groups in 100% of the animals, the rates of continued existence (animals were sacrificed till the body weight loss was found less than 25% from the starting experiment weight) variation. But, it was apparently noticed that the average survival time was 17 days for the JMAR animals, in comparison to all other animals which were dying by the end of the 23rd day of the trial. The tumor formation by both the cells was histologically distinct by the end of 31 days. It was also observed that one hundred percentages of the TU167 animals existed with negligible mass drop, apart from pathologically apparent and morphologically confirmed tongue tumors. Tumor formation caused by TU167 cells showed quite a lot of well-contained tumor layers, while JMAR tumors displayed an extraordinary spreading infiltrative development style. Further investigation by immunohistochemistry of tumor sections showed more positive and intense staining of S100A7 in JMAR bearing orthotopic tongue tumor as compared to TU167 (Fig. 1e). Taken together, our findings suggest that S100A7 is responsible for more tumorigenicity and likely to be anoikis resistance.

### Expression of the S100A7 in the human head and neck cancer specimens

We had immunostained tissue specimens of different malignant tumor regions of head and neck cancer specimens as well as a normal epithelium region with an anti-S100A7 rabbit antibody. Here, IHC sections of normal and tumor specimens (Fig. 2a) demonstrate that psoriasin is up-regulated in association with head and neck tumorigenesis. In the direction of exploring the significance of S100A7 in head and neck tumors, we studied whether S100A7 protein was changed in corresponding adjacent non-cancerous human epithelium and cancer tissue biopsy samples. As it is presented in Fig. 2b, S100A7 expression was elevated in 8 out of 12 tumor samples (66.66%) as evaluated with the neigh boring non-cancerous tissue, which illustrate either or no expression of S100A7. The loading control was used as β-actin for the blots that were used after reprobing. Psoriasin, protein expression was further evaluated by IHC in human tumor and normal oral tissue samples. The prevalence of S100A7 expression in these patients was 90.47% (38/42) as shown in Fig. 2c. Hence, we have analyzed ten normal oral samples for S100A7 expressions by IHC that shows negligible expression. A possible role of S100A7 in mediating invasion remains to be explored in future.

The article "Mechanistic attributes of S100A7 (psoriasin) in resistance of anoikis resulting tumor progression in squamous cell carcinoma of the oral cavity" was retracted in 2021. Reason: concerns about the images.

**Fig. 2:** Expression of S100A7 in the human head and neck tumor. **a** Representative immunohistochemical staining for S100A7 in tissues from normal and tumor sections. **b** Paired head and neck tumors (T) and adjacent normal (N) tissue were analyzed by immunoblotting with the indicated antibodies. **c** Immunohistochemical staining for S100A7 in tissues from normal and tumor sections in 42 samples and their correlation with tumorigenesis in table form.

### Secretion of the S100A7 protein in conditioned medium by anoikis resistant head and neck cancer cell and in saliva of head and neck cancer patients

To validate S100A7 as a biomarker for head and neck squamous cell carcinoma, S100A7 protein that got released in saliva by the patients or secreted in the conditioned medium by HNSCC cell lines were analyzed by Immunoblot. We had grown TU167 and JMAR cell in attached and detached condition. Later, condition medium containing equal amount of protein were immunoprecipitated and immunoblotted with S100A7 antibody. As shown in Fig. 3a, JMAR cell secreted S100A7 but not TU167 (anoikis sensitive cell line).We have also metabolically labeled the JMAR cells with [S35]-methionine and equal CPM from cell lysates and condition medium were immunoprecipitated with anti-S100A7 and separated by SDS-PAGE, further analysed by autoradiography (Fig. 3b). Next we have collected saliva samples from head and neck cancer patients as immunoblotting was performed for the detection of S100A7 protein expression. As shown in Fig. 3c, 18 out of 37 (48.65) saliva samples from the head and neck cancer patients has very high level of S100A7, and other has in the detectable range. Only 5 out of 37 (13.5%) tumor samples showed no expression of S100A7 in saliva, indicating that 32 out of 37 (86.5%) tumor samples showed expression of S100A7. On the other hand, we have analyzed four normal salivae, and S100A7 was absent in all four normal saliva samples. We were planning to examine more normal and head and neck cancer patient’s saliva for the detection of S100A7. Our present findings suggested that S100A7 can be utilized as novel protein biomarker for clinical diagnosis and disease status of head and neck cancer.

The article "Mechanistic attributes of S100A7 (psoriasin) in resistance of anoikis resulting tumor progression in squamous cell carcinoma of the oral cavity" was retracted in 2021. Reason: concerns about the images.

**Fig. 3:** S100A7 is secreted out in the medium by the cells and as well as in saliva by the head and neck cancer. **a** Conditioned medium from attached (24 h) TU167 and JMAR were immunoprecipitated by S100A7 antibody and immunoblotted with S100A7. **b** Cells are labelled with [35S]-methonine for 12 h in attach condition and cell lysates and condition medium containing equal CPM was immunoprecipitated with S100A7 antibody and analyzed by autoradiography. **c** Saliva from normal and head and neck cancer patient containing equal protein were analyzed by Western blot for the detection of S100A7.

### siRNA of S100A7 reverses anoikis resistant JMAR cells to anoikis sensitive cells

We have transfected anoikis resistant JMAR cells with siRNA of S100A7, control empty vector and Tu167 cells both were grown in attached or detached conditions for 1 or 2 days, and percentage of apoptotic cells were analyzed by flow cytometry. As shown in Fig. 4a, siRNA transfected JMAR cells underwent 39% apoptosis while only 14% cell death was observed in JMAR cells transfected with control vector after 24 h. After 48 h time point, 59% of JMAR cells transfected with siRNA showed apoptosis while only 12% of the control vector-transfected JMAR cells were apoptotic population. Apart from this 19% and 34% cell death were observed for 24 and 48 h respectively in the parental cell line TU167. Protein lysates from the same conditions were analyzed for the psoriasin expression by immunoblot. As shown in the Fig. 4b, S100A7 protein expression increased with the time interval, while it was down-regulated in detached JMAR cells transfected with siRNA.

**Fig. 4:** siRNA of S100A7 transfected cells can down-regulate the expression of S100A7 protein level through AKT signaling. **a** Flow cytometric analysis of sub G0/G1 cell population of JMAR and Tu167 cells. **b** Western blotting of S100A7 protein in JMAR cells transfected with siRNA of S100A7. The JMAR cell line was pre-incubated with or without LY294002 for 24 h in suspension culture prior to determination of apoptotic fraction of cells by flow cytometry. **c**, **d** Phosphorylation of Akt and expression of S100A7 by western blot.

### Up-regulation of S100A7 gene mediated by Akt phosphorylation signaling

To investigate whether cell detachment in anoikis resistant cell line directly initiates survival signaling, as well as to recognize its downstream molecules, protein kinase B (PKB; also known as AKT) activity was first examined, which helps to prevent the development of anoikis [34, 35]. Under detached conditions, Akt is activated in anoikis resistance JMAR cell line (Fig. 4d). This result also demonstrates that, S100A7 is up-regulated during cell detachment in anoikis resistance cell line that is mediated through the PKB survival pathway. This result, on the other hand, does not rule out the chance for the aggregate development which may further add to survival signaling in suspension. Significant PKB activation was observed in anoikis resistant cells. These phenomena suggested that PKB pathway promotes anoikis resistance via triggering of S100A7 action. Certainly, inhibition of PKB/PI3 K with specific agent LY294002 lead to inhibition of S100A7 mediated survival (Fig. 4c, d). From these observations, although it seems to be that PI3K/PKB signaling through S100A7 contributes to anoikis resistance, but more detailed understanding of the molecular mechanisms by which S100A7 contributes to anoikis resistance of human cells, is necessary in order to develop molecular targets that reverses anoikis resistant.

The article "Mechanistic attributes of S100A7 (psoriasin) in resistance of anoikis resulting tumor progression in squamous cell carcinoma of the oral cavity" was retracted in 2021. Reason: concerns about the images.

### S100A7 gene responsible for anoikis resistance in head and neck cancer

Further delineate the possible involvement of S100A7 in cancer cells, we have next established stable TU167 clones expressing different level of S100A7 (C1; clones expressing moderate level of S100A7, and C2; clones expressing higher level of S100A7) or control vector as observed by western and northern blot for the protein and RNA expression respectively (Fig. 5a, b). Later, we have also confirmed the expression of S100A7 protein by fluorescence microscopy (Fig. 5c). Next, we have grown the clones in both attached and detached condition for 1 or 2 days and percentages of apoptotic cells were analyzed by flow cytometry. As shown in Fig. 5d that stable clones of S100A7 were more anoikis resistant than the vector clones. Interestingly, we have observed that the C2 clones (higher level of S100A7) were more resistant towards apoptosis as in detached condition than C1 clones (moderate level of S100A7 expression), indicating the level of S100A7 as the quantitative indicator of developing anoikis resistance.

**Fig. 5:** Effect of S100A7 expression on anoikis in head and neck cancer cells. **a** Western blot analysis of vector and stable clones of S100A7 expression was moderate (C1) and higher (C2) level. The blot was reprobed with a β-actin as a loading control. **b** S100A7 mRNA expression in the stable clones. **c** Expression of S100A7 by immunofluorescence microscopy in the stable clones. **d** Detached cells were suspended in a 15 ml tube and rotated in the incubator at different time as described in the “Methods”, and flow cytometry assessed sub G0/G1 cells. Results shown are representative of three experiments.

The article "Mechanistic attributes of S100A7 (psoriasin) in resistance of anoikis resulting tumor progression in squamous cell carcinoma of the oral cavity" was retracted in 2021. Reason: concerns about the images.

### S100A7 gene responsible for tumorigenicity and metastatic potential in HNSCC

Here the probable reason of S100A7 expression for the growth features of HNSCC cells, which were calculated by the colony formation and cell proliferation rate. Over expression of S100A7 was escorted by a reproducible of the capability of cells to form outsized colonies in soft agar as differentiated with vector transfected control cells (Fig. 6a). Further assessment of the effect of choice for anoikis resistance on tumor development, it was calculated by the enlargement of the entire cell lines in an orthotopic tumor model [26]. In the subsequent experiment tumor formation and weight loss were observed in the athymic nude mice due to the tongues were injected with 1 × 106 vector/C1 and C2 (stable clones of S100A7) cells. Further all the animals i.e. 100% in all groups produced tumors, the rates of continued existence (animals were sacrificed till the body weight loss was found less than 25% from the starting experiment weight) variation was greatly observed. The midpoint survival for the C1 and C2 injected animals were 12 and 14 days respectively with all the animals dying at the end of the 25th day (Fig. 6b; Table 1). There was a significant difference between survival curve of both C1 (p < 0.0001) and C2 (p < 0.0001) with respect to the survival curve of mock-transfected TU167 clones injected in animals. Interestingly, there was also a significant difference (p < 0.0001) in the survival curve of orthotopic generated tumor mice injected with clones C1 and C2, that was analyzed by log-rank (Mantel-Cox) test. At the end of 25 days, hundred percentages of the mock-transfected TU167 injected animals were surviving with negligible mass loss, in spite of clinically obvious and histologically confirmed tumor lump. Since revealed in Fig. 6c, the lump produced by these cell lines were morphologically different. Tumor formation has taken place by the mock-transfected cells showing a number of controlled tumor colonies with minimal S100A7 staining while the C1 and C2 tumors confirmed a more diffusely infiltrative development model and over expression of S100A7. Together, these observations suggested that head and neck cancer cells expressing S100A7 have altered growth characteristics and tumorigenicity.

**Fig. 6:** Effect of S100A7 expression on Soft agar colony formation and tumorigenicity of head and neck cancer cells. **a** Anchorage independent growth of TU167 cells stably transfected with different level of S100A7 expression i.e. C1 and C2 clones along with vector-transfected. Results were representative photographs of soft agar colonies (n = 3). **b** Survival curve of nude mice orthotopically implanted with vector (pcDNA3.1) or S100A7 clones (C1 and C2) tumors. Nude mice were orthotopically implanted in the tongue with 1 × 10^6^ Vector or C1 or C2 S100A7 stable cells and observation showed weight loss with time. Animals losing more than 25% of their initial body weight were sacrificed. All the vector injected animals survived greater than 25 days without significant weight loss and therefore were sacrificed at that time point. **c** IHC of S100A7expression in FFPE tumor specimens from vector, C1, C2 orthotopically injected nude mice.

The article "Mechanistic attributes of S100A7 (psoriasin) in resistance of anoikis resulting tumor progression in squamous cell carcinoma of the oral cavity" was retracted in 2021. Reason: concerns about the images.

**Table 1:** Survival curve analysis using Kaplan–Meier survival test

TU167 clones	Median survival (day)	P value
pcDNA3.1	>25 or undefined	
C1 (moderate S100A7 expression)	14	<0.0001
C2 (high S100A7 expression)	12	<0.0001

Kaplan–Meier survival curve was plotted for three groups of mice receiving orthotropic tongue injection of (1) pcDNA3.1, (2) C1 and (3) C2 stable clones of TU167. *P* value was calculated by using log-rank (Mantel-Cox) test between mock (pcDNA3.1) vs. C1 or C2 groups.

## Conclusions

In summary, we provide new evidence that the S100A7 is responsible for anoikis resistance and tumorigenicity in human oral cancer cells and also positively controls the growth rate of the human head and neck cancer cells. This conclusion is based on the following facts: (1) up-regulation of S100A7 mRNA and protein in anoikis resistant cell lines; (2) Expression of the S100A7 in an orthotopic tumor model of SCCOC; (3) Expression of the S100A7 in human head and neck cancer; (4) Secretion of S100A7 protein in conditioned medium by anoikis resistant head & neck cancer cell and in saliva of head and neck cancer patients; (5) Up-regulation of S100A7 expression cells leads to an enhancement of the tumorigenicity and anchorage-independent growth of head and neck cancer cells; (6) S100A7 is up-regulated during cell detachment through Akt phosphorylation and finally, (7) S100A7 is responsible for anoikis resistance in head and neck cancer cells. The main goal is to screen cancer at an early stage so that adequate precautions can be done for further clinical intervention. In addition, the scrutinizing tool should be enough non-invasive and economical to allow extensive application. A material that gets secreted from tumor tissue, but not secreted by non-tumor, can easily and inexpensively measurable in saliva, serum or urine can act as a model biomarker, since the cancer is identified very precisely, early and non-invasive manner. Cancer is a varied illness, and it is very much doubtful that a sole biomarker will identify all types of cancer from a particular organ with high specificity and sensitivity. In fact, biomarker such as prostate-specific antigen (PSA) that claim to be highly sensitivity and tends to have little specificity as they do not identify cancer by itself however it is a more in common practice. We noted that a large mass population screening is a very high priority for maintaining high specificity (low false-positive rates). Still a minute false-positive rate interprets into a huge figure of populations subjected to pointless expensive diagnostic actions and mental tension. Therefore, biomarkers should be very much precise for cancer, and the application of quite a few such biomarkers of cancer would help the screening program very responsive and accurate. From our preliminary studies using immunohistochemistry and Western blotting of human oral cancer tumor and saliva specimens from cancer suffering patients and normal beings we have been noticed that a marker, S100A7 is being expressed in saliva, and tissues of oral cancer patients but almost absent in normal saliva and adjacent normal tissue. In a prospective clinical trial we will (1) measure the saliva levels of S100A7 in patients with oral leukoplakia treated with chemoprevention approaches prior to during and after therapy and determine whether there is any association between salivary S100A7 level and progression to oral cancer; and (2) measure the pre-treatment, immediate post-treatment and follow-up levels of salivary S100A7 to determine whether there is any association with the level of S100A7 and local recurrence. The molecular mechanisms, by which S100A7 affects the anoikis of human cells, were not still clear at the moment. Our findings have clearly demonstrated for the first time a potential role of S100A7 in anoikis and may be one of the early detection markers for head and neck cancer.

The article "Mechanistic attributes of S100A7 (psoriasin) in resistance of anoikis resulting tumor progression in squamous cell carcinoma of the oral cavity" was retracted in 2021. Reason: concerns about the images.

## Methods

### Reagents and cell line

TU167, JMAR, JMARC39, JMARC42 [33] and MDA-MB-468 human cancer cell lines were used. All cell lines were grown and maintained in DMEM medium supplemented with 10% fetal calf serum. For western blot analysis following primary and secondary antibodies were used: S100A7 (Imgenex Inc USA), β-actin (Sigma-Aldrich, St. Louis, MO), Akt and phospho Akt (Cell Signaling Technology, Danvers, MA) and anti- rabbit/mouse horseradish peroxidase-conjugated (Amersham, Piscataway, NJ).

### Generation of resistant cell line

TU167 cells were trypsinized and collected in a ventilated 15 ml centrifuge tube and incubated for 72 h on a revolving shaker with 5% CO_2_ at 37°C. The survived cells were cultured to 80–90% confluency, and a similar procedure was carried seven instances to produce the anoikis resistance JMAR cell line [36].

### Generation of stable cell line and transient transfection

The full-length coding sequence of psoriasin [GenBank: AJ012825.1] was cloned into pcDNA3.1 [37] and transfected into TU167 cells by Lipofectamine (Invitrogen, Burlington, ON, Canada). Stable clones were selected by zeocin, as a selection marker. Several clones were developed, and immunoblot determined protein expression of psoriasin. TU167-mock was generated by transfection with the empty vector. JMAR cells were also transfected with protein-specific siRNA (Qiagen, Mississauga, ON, Canada) of psoriasin. siRNA was conducted using Dharmafect-4 reagent (Dharmacon).

### Immunohistochemistry (IHC)

For Immunohistochemistry purpose, formalin-fixed tissue samples were embedded in paraffin followed by sectioning (5-µm) of the blocked tissue, which was collected from Department of Dentistry, Bankura Sammilani Medical College, approved by Institutional Ethical Committee [approval number: PR-HC/6-119/2895(8)] Bankura Sammilani Medical College, Bankura, West Bengal 722101. IHC was performed with appropriate primary anti-S100A7 antibody, positive and negative control was done simultaneously in the same experiments as previously described [38].

### Western blot and immuno-precipitation study

Protein was isolated from the cells using in NP-40 lysis buffer (Sigma-Aldrich, USA) for 60 min at 4°C. Proteins were separated in sodium dodecyl sulphate (SDS) polyacrylamide gel electrophoresis and transferred to nitrocellulose membrane. The Blocking of the Blots were done with Phosphate-buffered saline Tween (PBST) containing 3% bovine serum albumin for 1 h and subsequently incubated with the primary antibodies overnight at 4°C. After washing, blots were kept in secondary antibodies followed by development of bands by ECL reagents (Sigma-Aldrich, USA).The cells were metabolically labelled with 100 µCi/ml [35S]-methionine in methionine-free medium containing 2% dialyzed fetal bovine serum for 4–8 h. Cell extracts containing same trichloroacetic acid perceptible counts and immunoprecipitated by S100A7 antibody and resolved on SDS-PAGE and analyzed after exposure to film.

### Immunoblot analysis of human tissue and saliva

Human oral tissue and saliva specimens were collected from the Department of Dentistry, Bankura Sammilani Medical College, Bankura, West Bengal 722101 approved by Institutional Ethical Committee [approval number: PR-HC/6-119/2895(8)], Bankura Sammilani Medical College. All patients agreed to participate in this study and signed written informed consent. Tissue samples were homogenized in tissue lysis buffer (Sigma-Aldrich, USA) and proteins were isolated and examined by western blot analysis [39].

The article "Mechanistic attributes of S100A7 (psoriasin) in resistance of anoikis resulting tumor progression in squamous cell carcinoma of the oral cavity" was retracted in 2021. Reason: concerns about the images.

### Apoptosis assay

The determination of cell viability was done as described earlier [40]. Further, the flow cytometry was used to study the cell cycles (BD Corporation, Franklin Lakes, NJ, and USA) and the measurements of the apoptotic percentage were considered from sub-G0/G1 fraction. The data analysis was done by Cell Quest software version 2.0 (BD).

### Soft agar colony formation assay

The bi-layer of soft agar assay was executed by seeding cells (2 × 104 cells/well) which were suspended in 1 ml of 0.36% bacto-agar, Further the suspension with 1 ml was layered with 0.6% agar medium base layer in 12-well plates and the incubation of cells were done at 37°C with 5% CO_2_ for 3–4 weeks and needed every fifth day. After 14–21 days, colonies >0.05 mm were stained with crystal violet (0.005%) as described previously [41].

### Orthotopic animal model

Male athymic nude C57BL/6 mice of 6–10 weeks of age were accommodated in a particular pathogen-free animal facility, which were obtained from the All of the animal procedures were executed according to the guidelines approved by Department Of Biotechnology Institutional Animal Ethical Committee (approval no: E-1/MM-SMST/13), Indian Institute Of Technology, Kharagpur. Mice were divided into three groups (n = 10) namely pcDNA3.1, C1 (TU167 stably transfected with pcDNA3.1/S100A7 plasmid expressing intermediate level of S100A7), C2 (TU167 stably transfected with pcDNA3.1/S100A7 plasmid expressing high level of S100A7). The mouse received sub-mucosal injection of 1 × 106 of either mock (pcDNA3.1 empty vector) or pcDNA3.1/S100A7 plasmid expressing intermediate level of S100A7 or pcDNA3.1/S100A7 plasmid expressing high level of S100A7 stably transfected TU167 cells (suspended in a volume of 50 μl) directly into anterior tongue using a 1-ml syringe (Hamilton Co., Reno, Nevada) with a 30-gauge hypodermic needle. The injected animals were observed each alternative day for the growth of a lump on the tongue and mass loss were observed. CO2 inhalations were given for sacrificing the mice, when they had lost less than 25% of their pre-injection body weight [35].

### Kaplan–Meier survival analysis

Kaplan–Meier survival analysis of different clones of S100A7 in orthotopic tongue model was plotted using Graph Pad Prism 5.0, and log-rank (Mantel-Cox) test was applied to find out the statistical significance between the groups.

## Abbreviations

SCCOC: squamous cell carcinoma oral cavity
IHC: immunohistochemistry
ECM: extra cellular matrix
SCC: squamous cell cancer
SDS: sodium dodecyl sulphate
HNSCC: head and neck squamous cell carcinoma
FFPE: formalin-Fixed Paraffin Embedded
AKT (PKB): protein kinase B
